# Evaluation of the Inferior Vena Cava Diameter in Dehydrated Children Using Bedside Ultrasonography

**DOI:** 10.1155/2022/6395474

**Published:** 2022-08-24

**Authors:** Esra Akyüz Özkan, Mahmut Kılıç, Fatih Çalışkan, Ahmet Baydın

**Affiliations:** ^1^Ondokuz Mayıs University Medical Faculty, Department of Pediatrics, Samsun, Turkey; ^2^Yozgat Bozok University Medical Faculty, Department of Public Health, Yozgat, Turkey; ^3^Ondokuz Mayıs University Medical Faculty, Department of Emergency, Samsun, Turkey

## Abstract

**Objective:**

Bedside ultrasonography (US) is a new imaging modality that has begun to be used in the Pediatric Emergency Unit to evaluate inferior vena cava (IVC) diameter for intravascular volume status. In this article, we aimed to evaluate IVC diameter with bedside US before and after the fluid therapy in dehydrated children.

**Methods:**

A total of 124 dehydrated patients were enrolled, aged 8 months to 17 years. The maximum diameters of the IVC and aorta (AO) were measured. IVC/AO ratio and IVC collapsibility index IVC–CI were calculated before and after the fluid therapy and correlation with the degree of dehydration and laboratory parameters was investigated.

**Results:**

Of the 124 patients, 49.2% (*n* = 61) were male, the mean age was 7.5 ± 4.94 years. The IVC/AOs ratio was increased in mild and moderate/severe groups after fluid therapy compared to before fluid administration. While the mean rate of heart rate, blood urea nitrogen (BUN), creatinine, and uric acid values were higher in the moderate/severe group, potassium and HCO_3_ were lower. There was no significant change in AO diameter and IVC–CI after fluid therapy in all groups. When the factors affecting the IVC/AOs ratio were analyzed with the logistic regression backward model; the IVC/AO ratio was found to increase as the degree of dehydration decreased (Adj.*β* = −0.318) and as the age (Adj.*β* = 0.242) and CRP (Adj.*β* = 0.186) value increased.

**Conclusion:**

The IVC/AO ratio can be a promising index for the assessment and grading of dehydration in children, and cutoff values that vary according to age are necessary for a more objective assessment of dehydration.

## 1. Introduction

Dehydration is one of the most common causes of pediatric emergency department (PED) visits. According to a World Health Organization (WHO) report, acute diarrhea is responsible for approximately 17% of all pediatric deaths, making it the second most common cause of childhood death worldwide. A total of 1.8 million children under the age of 5 die from acute diarrhea each year. Diarrhea can cause dehydration, resulting in death [1].

Accurately assessing the degree of dehydration in children ensures the appropriate management of patients. Dehydration can lead to shock and even death if left undetected, and excessive fluid overload can cause heart failure, resulting in death [2].

No objective symptoms, clinical signs, or laboratory tests have demonstrated adequate sensitivity and specificity in dehydrated children [3]. Laboratory values can be used to assess the severity of dehydration; however, it is generally accepted that these parameters also have limited specificity and sensitivity [3]. In some studies by, WHO and the Centers for Disease Control and Prevention (CDC), clinical dehydration scales were found to be weak in determining the degree of dehydration [4–6]. A rapid, non-invasive, and objective assessment that accurately demonstrates volume status in dehydrated children is essential.

Central venous pressure (CVP) is considered to objectively assess intravascular volume. However, the insertion of a catheter for CVP is invasive, takes a long time, and is not routine, especially in pediatric patients. It may also predispose patients to thrombosis, infections, and arterial puncture [7].

Bedside ultrasonography (US) is a new imaging modality that has begun to be used in PEDs [8]. US evaluation of the inferior vena cava (IVC) has been used as a non-invasive diagnostic tool for intravascular volume evaluation [9]; it has been reported that CVP is correlated with IVC diameter in dehydrated children [10].

In the literature, patients with dehydration or sepsis have been evaluated using the IVC index (IVC/Aorta (AO)) and the IVC collapsibility index (IVC–CI), and it has been suggested that these indices provide information easily and objectively [7, 8, 11]. In some studies, it was observed that these indices were not affected by age or body surface area (BSA) in dehydrated children, while some other publications showed an increase with age in healthy children [12]. In the literature, IVC/AOs was found to be more reliable than IVC-CI and various cutoff values were given [13, 14].

We investigated the changes in these two indices before and after intravenous fluid administration in patients who presented to the PED with dehydration due to diarrhea or vomiting. In addition, we aimed to group patients as mild, moderate or severe, to correlate their severity levels with these indices and to find an objective cutoff value for mild dehydration. We also aimed to examine the correlation of these indices with laboratory tests and vital signs of the patients, as well as their ages and their BSAs.

## 2. Materials and Methods

### 2.1. Study Design

This prospective, observational study was conducted in the PED from June 2021 to October 2021 at Ondokuz Mayıs University Faculty of Medicine, a tertiary care hospital. Ethics committee approval was obtained for the study from the Institutional Review Board (OMU KAEK 2021/282). Informed written consent was obtained from the parents of each subject.

### 2.2. Participant Selection

A total of 124 children aged from 8 months to 17 years presenting with vomiting or diarrhea and with a clinical evidence of dehydration needing IV fluid administration, as determined by the attending pediatric emergency physician, were considered as subjects. Children with a history of congenital heart disease and heart failure, hemodialysis patients, children with acute blood loss and connective tissue disease and patients on mechanical ventilation were excluded from the study.

The grading of dehydration was performed as follows by the attending clinician, who was blinded to the results of the ultrasound;

- Mild dehydration; increased or normal heart rate, normal physical signs of thirst, and decreased urine output,
- Moderate dehydration; tachycardia, irritable or lethargy, decreased urine output, sunken eyes and fontanel, decreased tears, low skin turgor, dry mucous membranes, delayed capillary filling (>1.5 s), coldness and pallor,
- Severe dehydration; no or rapid weak peripheral pulse, decreased blood pressure, no urine output, very sunken eyes and fontanel, dried mucous membranes, low skin turgor, no tears, cold and mottled skin, depressed consciousness, very delayed capillary filling (>3 s) [15].

### 2.3. Sample Size

The sample size was calculated using the *G* power 3.1 programs. In the sample size calculation, 11 factors were assumed, to affect the IVC/AO ratio. These were; pulse, diastolic blood pressure (DBP), systolic blood pressure (SBP), blood urea nitrogen (BUN), HCO_3_, C-reactive protein (CRP), uric acid, creatinine, potassium (K), degree of dehydration (ordinal) and age. Accordingly, to analyze the impact of at least 11 factors on the IVC/AO ratio using linear regression, the minimum sample size (power 1− *β* = 0.90) was calculated as *n* = 82 when the effect size was taken as *R*2 = 0.30 and the margin of error as *α* = 0.05.

### 2.4. Measurements

History and physical examination, demographic parameters (age and gender), height, weight, body mass index (BMI), and BSA were recorded along with the clinical grading of dehydration. BMI was calculated by dividing weight by height in meters squared and BSA was calculated by Mosteller's formula [15].

The vital signs (temperature, pulse, blood pressure) of the patients were evaluated and laboratory tests were taken to determine complete blood count (CBC), uric acid, creatinine, BUN, glucose, sodium (Na), K, CRP, HCO_3_, and lactate. Bedside US of all patients were performed by the same person (an emergency specialist with a US certificate) who was blinded to the patients' clinical and laboratory parameters, before and immediately after fluid administration. All dehydrated subjects received the same quantities of IV fluids (20 cc/kg 0.9% isotonic, maximum 500 cc).

### 2.5. Ultrasound Protocol

The patients were scanned by bedside US (GE Logic-E ultrasound machine, 4C RS convex array probe in the 2–5 mHz range) while lying in the supine position. After the gel was applied, the probe was placed longitudinally on the patient's abdomen on the midline, 1 cm away from the xiphoid process during normal breathing and the intrahepatic segment of IVC was examined. The probe was then oriented in the transverse plane; both the IVC and the upper abdominal aorta were visible at this point above the vertebral trunk shadow, just caudal to the insertion of the left renal vein into the IVC. The maximum anterior-posterior IVC diameter and descending AO diameter were measured and the IVC/AOs ratio was calculated for the AOs (IVC/AOs) [16, 17]. The maximum IVC diameter was obtained during the expiratory phase of the respiratory cycle, while the maximum AO diameter was obtained during the systolic phase of the cardiac cycle. Both measurements were performed in the transverse plane and in the B-mode US.

The probe was then turned longitudinally, centered 2–3 cm below the point where the IVC entered the right atrium and confluence of the hepatic veins. The maximum expiratory and minimum diameters in the M-mode (IVC min, IVC max) of the IVC were then recorded, taking care to align perpendicular to the anterior and posterior walls of the IVC. A measurement close to the transverse view of the left portal vein was obtained in all patients [12]. IVC-CI, defined as 100x (IVC max-IVC min)/IVC max was then recorded.

### 2.6. Statistical Analysis

For the analysis of the data, version 25.0 of IBM SPSS (Statistical Package for the Social Sciences) was used. Shapiro–Wilk test and histogram were used to examine the normal distribution suitability of the variables. Descriptive statistics were presented as mean (±) standard deviation. The significance of differences between groups in terms of averages was assessed by the following tests; Kruskal-Wallis test, One way ANOVA, Pearson correlation, Spearman Rho, and paired samples *t*-test. The degree of dehydration of the patients was classified as mild, moderate and severe by the clinician according to their clinical status. Since the number of patients with severe dehydration was low, they were combined with the moderate group. Variables that were found to be significant at *p* < 0.2 in the correlation and ANOVA tests were analyzed in multivariate linear regression (LR) using the backward model. Results for *p* < 0.05 were considered statistically significant. Receiver operating characteristic (ROC) analysis was performed to predict the degree of dehydration of the IVC/AOs ratio value. ROC analysis was used to determine the cutoff value of mild and moderate-severe dehydration and its sensitivity and selectivity in estimation.

## 3. Results

This study included 124 children who had been treated for diarrhea or vomiting, and 62.9% (*n* = 78) of them had mild dehydration symptoms, 37.1% (*n* = 37) had moderate dehydration symptoms, and 7.3% (*n* = 9) had severe dehydration symptoms. Additionally, 49.2% (*n* = 61) of the children (*n* = 124) were male. The age range was between 8 months and 17 years, and the mean age was 7.5 ± 4.94 years.

The patients were categorized into three groups based on their degree of dehydration: mild, moderate, and severe. It was discovered that their age, BMI percentile, IVC-CI, aortic diameter, minimum and maximum IVC diameters, and SBP, DBP, Na, glucose, hemoglobin (Hb), hematocrit (Htc), pH, lactate, and CRP levels were not statistically different (*p* > 0.05).

The moderate and severe groups had statistically lower IVC/AO and IVC transverse diameters than the mild group both before and after fluid therapy. Although the moderate and severe groups had higher mean heart rate per minute, BUN, creatinine, and uric acid values, their K and HCO_3_ values were lower (Table 1).

The IVC/AO diameters were measured before and after fluid administration. The mild, moderate, and severe groups exhibited a statistically significant increase in IVC/AO ratio values after fluid therapy.  Figure 1 depicts the IVC/AO ratios before and after fluid therapy based on the degree of dehydration.

The mild, moderate, and severe groups did not exhibit a statistically significant difference in aortic diameter and IVC-CI values after fluid therapy (Table 2). There was a positive correlation between the IVC/AO ratio and age, BSA, DBP, SBP, HCO3, and CRP, as well as a statistically significant negative correlation with the degree of dehydration (*r* = −0.348) and heart rate (*r* = −0.190). There was no significant correlation between the IVC/AO ratio and the white blood cell (WBC), Hb, Htc, glucose, BUN, creatinine, uric acid, Na, K, pH, and lactate levels (Table 3).

When the factors affecting the IVC/AO ratio were analyzed using the LR backward model, the IVC/AO ratio was found to increase as the degree of dehydration decreased (Adj.*β* = −0.318) and as the age (Adj.*β* = 0.242) and CRP (Adj.*β* = 0.186) value increased. These three variables represented 17.7% (Adj.*R*^2^ = 0.177) of the total change in the IVC/AO ratio. The weight, BSA, pulse, DBP, SBP, BUN, uric acid, creatinine, HCO_3_, K, and lactate levels were not statistically significant in the LR analysis (Table 4).

The IVC–CI was found to have no difference based on the degree of dehydration and no significant correlation with the other variables. In addition, the ROC analysis revealed that the IVC-CI could not be used as a predictor of the degree of dehydration (the area under the curve (AUC) value was 0.515 (95% CI; 0.408–0.623); *p*=0.774).

When the ROC analysis was used to examine if the IVC/AOs ratio could be used to predict the degree of dehydration to detect mild dehydration (AUC value: 0.706 (95% CI; 0.605–0.808); *p* < 0.001), the cutoff value was found to be ≤ 1.0284 (sensitivity: 71.8%; specificity: 63.0%) (Figure 2). Although children under 5 years old had a cutoff value of 0.9641 (sensitivity: 79.3%; specificity: 68.2%), children over 5 years old had a cutoff value of 1.0987 (sensitivity: 65.3%; specificity: 62.5%).

## 4. Discussion

The literature has demonstrated that ultrasound (US) could be used to diagnose severe dehydration in children with diarrhea [7]. Previous studies have shown that measuring the IVC diameter with the US can be used as an indicator to evaluate the volume status in dehydrated patients [7–9]. IVC diameter measurement with the US is an early predictor of shock in trauma patients and a useful method for measuring volume status in septic and hypotensive patients in intensive care units [18].

The IVC of dehydrated patients was evaluated using two indexes in the literature: the IVC/AO ratio and IVC–CI. This study aimed to evaluate the use of US in diagnosing and grading dehydration before and after fluid therapy, and both indexes were used to improve the objectivity and reliability of assessing dehydrated children. It also aimed to determine the clinical and laboratory parameters that affect the IVC/AO ratio and the IVC–CI.

The findings suggested that the IVC diameter decreased as the degree of dehydration increased and that it increased after fluid therapy, whereas the AO diameter remained unchanged. Chen et al. [19] discovered that the AO diameter did not change after fluid therapy, which is consistent with our results. Although the IVC diameter has been shown in the literature to decrease as the degree of dehydration increases, it cannot be used without nomograms to diagnose children in clinical practice [7].

Adewumi et al. [7] suggested that the abdominal aortic diameter, similar to the IVC diameter, has a correlation with BSA, age, and gender and that there is no statistically significant change in the aortic size with hydration status. Therefore, they suggested that the IVC/AO ratio could be used without nomograms to calculate the BSA for each age group. In this study, there was a positive correlation between the IVC/AO ratio and age, and contrary to the findings of Adewumi et al. [7], the IVC/AO ratio increased with age. Similar to this study on normal hydrated children, the study by Mannarino et al. [12] demonstrated that the IVC/AO ratio increased as the age and BSA increased, suggesting that the IVC/AO ratio showed age-related values, which were 0.83 and 1.22 for children under the age of 1 and children above the age of 1, respectively. Although the literature has suggested that the IVC/AO ratio does not change with age in dehydrated patients, no publication with a statistical evaluation has been found [7]. Although the correlation analysis in our study revealed a positive correlation between the BSA and IVC/AO ratio, the regression analysis revealed that the BSA did not affect the IVC/AO ratio.

There was a positive correlation between the CRP and IVC/AO ratio in this study. The literature has demonstrated that high CRP levels are associated with diastolic dysfunction and heart failure risk [20]. The IVC/AO ratio in heart failure patients increases because of volume overload. Therefore, the positive correlation between the IVC/AO ratio and CRP is reasonable, as CRP also increases in heart failure patients. Kim et al. [21] conducted a study on 423 adults with septic shock, and non-survivors were discovered to have a higher mean IVC diameter ratio than survivors. The IVC diameter ratio was greater than 1.31 and was associated with in-hospital mortality (sensitivity: 75% and specificity: 42%). CRP values have also been found to be positively correlated with mortality [22].

Although the IVC/AO ratio in all patients in the mild, moderate, and severe groups statistically increased significantly before and after fluid therapy, there was no such a correlation for the IVC–CI in this study. Additionally, although the correlation analysis revealed a significant inverse correlation between the IVC/AO ratio and the degree of dehydration, there was no correlation in the IVC–CI. Studies that have compared the IVC/AO ratio with the IVC–CI have concluded that the IVC/AO ratio is a valuable and superior alternative to the IVC–CI [13, 14]. However, some studies have also revealed a correlation between CVP and IVC–CI in dehydrated or septic patients [10, 11]. Long et al. [22] discovered no correlation between the IVC–CI and fluid responsiveness in children with sepsis. Babaie et al. [23] investigated the correlation between CVP and IVC sonographic indexes and demonstrated that the IVC–CI was 45.5% sensitive and 91.7% specific, with a positive predictive value of 71.4 and a negative predictive value of 78.6 for predicting CVP <8; the sensitivity and specificity of IVC/AO ratio were 50.8% and 87.5% respectively, with a positive predictive value of 64.7 and a negative predictive value of 79.2 for predicting CVP <8.

The IVC/AO ratio can be measured longitudinally and transversely using B-mode US [7, 19]. In this study, this ratio was measured using B-mode US in the transverse plane. Durajska et al. [24] measured the IVC/AO ratio in the transverse and longitudinal planes and demonstrated that the two measurements had similar results and may be used interchangeably to assess the hydration status of patients.

In this study, the mild, moderate, and severe groups had IVC/AO ratios of 1.17 ± 0.22, 1.03 ± 0.26, and 0.95 ± 0.27, respectively, and these ratios increased statistically after fluid therapy. Chen et al. [19] reported that the IVC/AO ratio was 0.75 in patients but 1.01 in the control group measured using B-mode US and transverse plane. In another study by Adewumi et al. [7]; the mean IVC/AOs was 0.75 ± 0.07 for mild, 0.55 ± 0.07 for moderate and 0.33 ± 0.05 for severe dehydration using B-mode US and longitudinal plane and found an inverse correlation between IVC/AOs and dehydration degree.

In this study, the cutoff values were 0.96 for children under 5 years old (sensitivity: 79.3%; specificity: 68.2%) and 1.09 (sensitivity: 65.3%; specificity: 62.5%) for children over 5 years old. Values below this level indicate moderate/severe dehydration, while those above this level indicate mild dehydration. We could not determine a suitable cutoff value for all age groups owing to the insufficient number of patients in this study. Chen et al. [19] obtained a cutoff value of 0.72 with 100% sensitivity and 39% specificity measuring with the B-mode US and transverse plane. In another study, the IVC/AO cutoff value of 0.8 was demonstrated with a sensitivity of 86% and a specificity of 56% for diagnosing significant dehydration using B-mode US and transverse plane [17]. Adewumi et al. [7] showed 0.86 with 96% sensitivity, and 96% specificity. Levine et al. [13] found 1.22 cutoff values for severe dehydration with 93% sensitivity and 59% specificity using B-mode US and longitudinal plane.

### 4.1. Study Limitations

Since there were insufficient numbers of patients in each age group, the cutoff value for the IVC/AO ratio could not be determined by age. The other limitations are being single center, the US being performed by a single sonographer, and the lack of a control group.

In conclusion, the IVC/AO ratio may be an objective index for assessing dehydration and can be used routinely to classify the degree of dehydration in clinical settings. Although the IVC/AO ratio had a correlation with the degree of dehydration and increased with fluid therapy, the IVC–CI exhibited no such correlation. Contrary to the findings in the literature, the IVC/AO ratio increased with age; thus, age-standardized cutoff values should be adapted to the degree of dehydration in children for a more objective evaluation. Therefore, the age-specific cutoff values for the IVC/AO ratio should be evaluated in future studies.

## Figures and Tables

**Figure 1:** The values of IVC/AOs before and after fluid therapy according to the degree of dehydration.

**Figure 2:** Receiver operator characteristic (ROC) curve of IVC/AO ratio to identify the degree of dehydration is mild.

**Table 1:** Comparison of the demographic characteristics, cardiac and biochemical parameters according to the degree of dehydration

Variables	Dehydration degree								
	Mild (*n* = 78)		Moderate (*n* = 37)		Severe (*n* = 9)		Total (*n* = 124)		
	Mean	SD	Mean	SD	Mean	SD	Mean	SD	ANOVA *p* value
Age (year)	7.55	4.50	7.16	5.66	8.05	5.90	7.47	4.94	0.867
Weight persentil (%)	60.15	30.35	48.82	34.13	38.30	29.76	55.18	32.00	**0.052**
BMI persentil (%)	65.93	34.16	61.23	33.73	47.37	33.75	63.18	34.08	0.279
IVC/AO first^a^	1.1712	0.2265	1.0352	0.2647	0.9542	0.2733	1.1149	0.2516	**0.003**
IVC/AO last^b^	1.4157	0.2386	1.2689	0.2764	1.1608	0.1275	1.3547	0.2589	**0.015**
IVC trans First^a^ (mm)	1.1664	0.3799	0.8986	0.3566	0.8711	0.2973	1.0650	0.3885	**0.001**
IVC trans Last^b^ (mm)	1.4602	0.3290	1.2066	0.4405	1.2260	0.4082	1.3610	0.3898	**0.012**
AO first (mm)^a^	0.9959	0.2547	0.8822	0.3045	0.9656	0.4127	0.9598	0.2854	0.136
AO last (mm)^b^	1.0427	0.2259	0.9782	0.2716	0.9175	0.1733	1.0152	0.2405	0.372
IVC-CI first^a^	24.98	10.42	24.41	10.62	22.87	12.21	23.50	10.21	0.841
IVC-CI last^b^	23.29	10.14	22.83	9.46	29.28	15.13	24.65	10.54	0.429
IVC min first^a^ (mm)	0.6001	0.1601	0.6143	0.2288	0.6706	0.3137	0.6095	0.1952	0.586
IVC min last^b^ (mm)	0.6518	0.1803	0.6200	0.2010	0.5320	0.1359	0.6340	0.1858	0.348
IVC max first^a^ (mm)	0.8042	0.1979	0.8238	0.3269	0.8581	0.3434	0.8140	0.2524	0.802
IVC max last^b^ (mm)	0.8559	0.2386	0.8093	0.2394	0.7980	0.3615	0.8366	0.2445	0.674
Pulse (/minute)	98.46	11.31	103.27	13.37	108.78	24.76	100.65	13.50	**0.040** ^*∗*^
DBP (mmHg)	63.38	5.98	62.24	5.48	62.78	8.33	63.00	6.00	0.640
SBP (mmHg)	98.27	8.75	96.43	11.00	95.56	12.10	97.52	9.68	0.525
Glucose (mg/dL)	97.18	16.39	97.51	29.97	92.33	42.10	96.91	23.38	0.824^*∗*^
Bun (mg/dL)	12.64	3.63	15.78	4.48	24.58	14.00	14.45	6.13	**0.001** ^*∗*^
Creatinine(mg/dL)	0.48	0.13	0.50	0.17	0.84	0.44	0.53	0.37	**0.029** ^*∗*^
Uric acid (mg/dL)	4.25	1.10	4.87	1.38	7.26	2.86	4.67	1.58	**0.002** ^*∗*^
Na (mEq/L)	136.86	2.38	137.46	3.29	137.00	3.46	137.04	2.75	0.566
K (mEq/L)	4.23	0.31	4.11	0.36	3.71	0.65	4.16	0.38	**<0.001**
WBC (/uL)	11.04	3.72	11.56	4.35	13.20	6.83	11.36	4.19	0.722^*∗*^
Hb (g/dL)	13.06	1.24	12.91	1.85	13.09	1.97	13.18	2.04	0.872
HTC (%)	37.21	3.43	37.23	5.20	38.46	6.52	37.67	4.98	0.708
pH	7.40	0.039	7.40	0.06	7.35	0.12	7.40	0.06	0.248^*∗*^
HCO3 (mmol/L)	22.05	1.74	20.84	3.05	19.50	6.38	21.50	2.82	**0.056** ^*∗*^
Lactate (mmol/L)	1.55	0.46	1.89	0.78	2.38	1.56	1.71	0.71	0.102^*∗*^
CRP (mg/L)	9.26	16.97	8.05	19.18	25.07	48.07	10.0952	21.4623	0.119^*∗*^

^*∗*^ Kruskal-Wallis H. SD: Standard Deviation. AO: Aorta, IVC: Inferior vena cava, CI: Collapsibility index BMI: Body mass index, DBP: Diastolic blood pressure, SBP: Systolic blood pressure, BUN: Blood Urea Nitrogen, Na: sodium, K: potassium, WBC: white blood cell, Hb: hemoglobin, Htc: hematocrit, CRP: C-reactive protein.^a^ before fluid therapy.^b^ after fluid therapy.

**Table 2:** Comparison of sonographic parameters before and after fluid therapy.

Cardiac parameters	Mild (*n* = 52)			Moderate and severe (*n* = 33)			Total (*n* = 85)		
	Mean			Mean			Mean		
	First	After	Sig.^*∗*^	First	After	Sig.^*∗*^	First	After	Sig.^*∗*^
IVC/AO	1.1558	1.4157	**0.000**	0.9983	1.2554	**0.000**	1.0958	1.3547	**0.000**
IVC transverse (mm)	1.1693	1.4602	**0.000**	0.8741	1.2094	**0.000**	1.0526	1.3610	**0.000**
AO (mm)	1.0173	1.0427	0.371	0.9009	0.9706	0.136	0.9730	1.0152	0.089
IVC min (mm)	0.5984	0.6518	**0.020**	0.5570	0.6067	0.077	0.5821	0.6340	**0.003**
IVC max (mm)	0.8112	0.8559	**0.053**	0.7653	0.8076	0.143	0.7928	0.8366	**0.014**
IVC-CI	25.74	23.29	0.186	26.16	23.81	0.320	23.50	25.91	0.095

^*∗*^Paired *t*-test. AO: Aorta, IVC: Inferior vena cava, CI: Collapsibility index.

**Table 3:** Correlation between IVC, AO diameter, laboratory parameters and vital signs.

	IVC/AO first^a^	IVC-CI_First^a^	VCI transverse (mm)	AO (mm)	IVC min (mm)	IVC max (mm)	Age (yr)	Weight percentil (%)	BSA	Pulse (/minute)	DBP (mmHg)	SBP (mmHg)	WBC (/uL)	Hb (g/dL)	HTC (%)
IVC/AO first^a^	1														
IVC-CI_First^a^	−0.015	1													
IVC transvers (mm)	**0.600** ^*∗∗*^	0.084	1												
AO (mm)	−0.069	0.157	**0.731** ^*∗∗*^	1											
IVC min (mm)	**0.286** ^*∗∗*^	**−0.304** ^*∗∗*^	**0.542** ^*∗∗*^	**0.431** ^*∗∗*^	1										
IVC max (mm)	**0.286** ^*∗∗*^	0.145	**0.595** ^*∗∗*^	**0.521** ^*∗∗*^	**0.890** ^*∗∗*^	1									
Age (yr)	**0.254** ^*∗∗*^	0.142	**0.647** ^*∗∗*^	**0.620** ^*∗∗*^	**0.607** ^*∗∗*^	**0.693** ^*∗∗*^	1								
Weight percentil (%)	0.052	−0.032	0.164	**0.186** ^*∗*^	0.039	0.005	−0.049	1							
BSA	**0.245** ^*∗∗*^	0.124	**0.670** ^*∗∗*^	**0.651** ^*∗∗*^	**0.599** ^*∗∗*^	**0.671** ^*∗∗*^	**0.946** ^*∗∗*^	**0.195** ^*∗*^	1						
Pulse (/minute)	**−0.190** ^*∗*^	−0.144	**−0.522** ^*∗∗*^	**−0.541** ^*∗∗*^	**−0.339** ^*∗∗*^	**−0.427** ^*∗∗*^	**−0.666** ^*∗∗*^	−0.015	**−0.648** ^*∗∗*^	1					
DBP (mmHg)	**0.199** ^*∗*^	0.020	**0.501** ^*∗∗*^	**0.446** ^*∗∗*^	**0.367** ^*∗∗*^	**0.384** ^*∗∗*^	**0.632** ^*∗∗*^	−0.081	**0.569** ^*∗∗*^	**−0.450** ^*∗∗*^	1				
SBP (mmHg)	**0.237** ^*∗∗*^	0.128	**0.635** ^*∗∗*^	**0.618** ^*∗∗*^	**0.479** ^*∗∗*^	**0.549** ^*∗∗*^	**0.804** ^*∗∗*^	−0.031	**0.746 ** ^*∗∗*^	**−0.535** ^*∗∗*^	**0.741** ^*∗∗*^	1			
WBC (/uL)	0.011	0.078	−0.070	−0.085	0.090	0.114	0.076	0.004	0.090	0.029	0.117	0.057	1		
Hb (g/dL)	0.111	**0.196** ^*∗*^	**0.355** ^*∗∗*^	**0.389** ^*∗∗*^	**0.373** ^*∗∗*^	**0.478 ** ^*∗∗*^	**0.488** ^*∗∗*^	**0.267** ^*∗∗*^	**0.552** ^*∗∗*^	**−0.341** ^*∗∗*^	0.175	**0.345 ** ^*∗∗*^	**0.184** ^*∗*^	1	
HTC (%)	0.079	0.168	**0.247** ^*∗∗*^	**0.276** ^*∗∗*^	**0.324** ^*∗∗*^	**0.409** ^*∗∗*^	**0.454** ^*∗∗*^	**0.258** ^*∗∗*^	**0.516** ^*∗∗*^	**−0.228** ^*∗*^	0.146	**0.300 ** ^*∗∗*^	**0.181** ^*∗*^	**0.919** ^*∗∗*^	1
	*IVC/AO*	*IVC CI*	*IVC transverse (mm)*	*AO (mm)*	*IVC min (mm)*	*IVC max (mm)*	*Glucose (mg/dL)*	*BUN (mg/dL)*	*Creatinine (mg/dL)*	*Uric acid (mg/dL)*	*Na (mEq/L)*	*K (mEq/L)*	*pH*	*HCO *_*3*_ * (mmol/L)*	*Lactate (mmol/L)*
Glucose (mg/dL)	0.113	0.098	**0.240** ^*∗∗*^	**0.229** ^*∗*^	**0.193** ^*∗*^	**0.254** ^*∗∗*^	1								
BUN (mg/dL)	−0.104	−0.100	**−0.200** ^*∗*^	−0.174	−0.046	−0.122	0.028	1							
Creatinine (mg/dL)	0.161	−0.003	**0.319** ^*∗∗*^	**0.266** ^*∗∗*^	**0.430** ^*∗∗*^	**0.434** ^*∗∗*^	0.328^*∗∗*^	0.503^*∗∗*^	1						
Uric acid (mg/dL)	−0.082	0.038	−0.139	−0.135	0.024	0.027	−0.235^*∗*^	0.521^*∗∗*^	0.409^*∗∗*^	1					
Na (mEq/L)	−0.073	0.158	0.015	0.088	0.010	0.066	0.356^*∗∗*^	0.101	0.177	0.022	1				
K (mEq/L)	−0.045	0.125	−0.007	0.039	−0.003	0.048	0.084	−0.296^*∗∗*^	−0.230^*∗*^	−0.059	0.238^*∗∗*^	1			
pH	0.049	−0.075	0.177	**0.206** ^*∗*^	0.057	0.045	0.170	−0.249^*∗∗*^	−0.132	−0.251^*∗∗*^	−0.259^*∗∗*^	−0.020	1		
HCO_3_ (mmol/L)	**0.206** ^*∗*^	−0.019	**0.377** ^*∗∗*^	**0.332** ^*∗∗*^	**0.272** ^*∗∗*^	**0.267** ^*∗∗*^	0.428^*∗∗*^	−0.238^*∗∗*^	0.071	−0.340^*∗∗*^	0.012	0.150	0.672^*∗∗*^	1	
Lactate (mmol/L)	−0.052	0.104	−0.079	0.007	0.046	0.101	0.008	0.154	0.122	0.124	−0.012	−0.196^*∗*^	−0.063	−0.225^*∗*^	1
CRP (mg/L)	**0.202** ^*∗*^	−0.024	0.137	−0.001	**0.290** ^*∗∗*^	**0.275** ^*∗∗*^	0.058	0.136	0.334^*∗∗*^	0.108	−0.054	−0.177	−0.222^*∗*^	−0.098	0.134
Dehydration degree	**−0.348** ^*∗∗*^	−0.030	**−0.385** ^*∗∗*^	−0.229^*∗*^	−0.016	−0.055	−0.044	**0.356** ^*∗∗*^	0.143	0.**308**^*∗∗*^	0.050	**−0.258** ^*∗∗*^	−0.105	−0**.215**^*∗*^	0.**193**^*∗*^

^*∗∗*^. Correlation is significant at the 0.01 level (2-tailed). ^*∗*^. Correlation is significant at the 0.05 level (2-tailed). AO: Aorta, IVC: Inferior vena cava, CI: Collapsibility index BSA: Body surface area, DBP: Diastolic blood pressure, SBP: Systolic blood pressure, BUN: Blood Urea Nitrogen, WBC: white blood cell, Hb: hemoglobin, Htc: hematocrit.^a^ before fluid therapy. †: Non-parametric Spearman Rho correlations. AO: Aorta, IVC: Inferior vena cava, CI: Collapsibility index, BUN: Blood Urea Nitrogen, Na: sodium, K: potassium, CRP; C-reactive protein.

**Table 4:** Linear regression analysis of factors that effecting IVC/AO ratio.

Adj.*R*^2^ = 0.177	Unstandardized coefficients		95.0% confidence interval for B		Standardized coefficients	*t*	Sig.
	B	Std. Error	Lower bound	Upper bound	*β*		
(Constant)	1.179	0.063	1.054	1.303		18.740	0.000
Age	0.012	0.004	0.004	0.021	0.242	2.786	**0.006**
C-reactive protein	0.002	0.001	0.000	0.004	0.186	2.124	**0.036**
Dehydration degree	−0.130	0.035	−0.198	−0.061	-0.318	−3.739	**0.000**

a. Independent Variables: age, body surface area, Pulse, diastolic blood pressure, systolic blood pressure, BUN, uric acid, creatinine, HCO3, C-reactive protein, potassium, lactate, dehydrated degree (ordinal).

## Data Availability

The data used to support the findings of this study are available from the corresponding author upon request.

## References

[1] World Health Organization (2005). *World Health Report 2005: Making Every Mother and Child Count: Statistical Annex3*.

[2] Holliday M. A., Friedman A. L., Segar W. E., Chesney R., Finberg L. (2004). Acute hospital-induced hyponatremia in children: a physiologic approach. *The Journal of Pediatrics*.

[3] Steiner M. J., DeWalt D. A., Byerley J. S. (2004). Is this child dehydrated?. *JAMA*.

[4] Levine A. C., Munyaneza R. M., Glavis-Bloom J. (2013). Prediction of severe disease in children with diarrhea in a resource-limited setting. *PLoS One*.

[5] Jauregui J., Nelson D., Choo E. (2014). External validation and comparison of three pediatric clinical dehydration scales. *PLoS One*.

[6] Kinlin L. M., Freedman S. B. (2012). Evaluation of a clinical dehydration scale in children requiring intravenous rehydration. *Pediatrics*.

[7] Idowu B., Adewumi A., Braimoh K., M Adesiyun O., Ololu-Zubair H. (2019). Correlation of sonographic inferior vena cava and aorta diameter ratio with dehydration in Nigerian children. *Nigerian Journal of Clinical Practice*.

[8] Chen L., Baker M. D. (2007). Novel applications of ultrasound in pediatric emergency medicine. *Pediatric Emergency Care*.

[9] Pershad J., Myers S., Plouman C. (2004). Bedside limited echocardiography by the emergency physician is accurate during evaluation of the critically ill patient. *Pediatrics*.

[10] Karacabey S., Sanri E., Guneysel O. (2016). A non-invasive method for assessment of intravascular fluid status: inferior vena cava diameters and collapsibility index. *Pakistan Journal of Medical Sciences*.

[11] Sawe H. R., Haeffele C., Mfinanga J. A., Mwafongo V. G., Reynolds T. A. (2016). Predicting fluid responsiveness using bedside ultrasound measurements of the inferior vena cava and physician gestalt in the emergency department of an urban public hospital in sub-saharan africa. *PLoS One*.

[12] Mannarino S., Bulzomì P., Codazzi A. C. (2019). Inferior vena cava, abdominal aorta, and IVC-to-aorta ratio in healthy Caucasian children: ultrasound Z-scores according to BSA and age. *Journal of Cardiology*.

[13] Levine A. C., Shah S. P., Umulisa I. (2010). Ultrasound assessment of severe dehydration in children with diarrhea and vomiting. *Academic Emergency Medicine*.

[14] Sridhar H., Mangalore P., Chandrasekaran V. P. (2012). Caval aorta index and central venous pressure correlation in assessing fluid status! Ultrasound bridging the gap. *Journal of Emergency Medicine*.

[15] Greenbaum L. A. (2011). Nelson textbook of paediatrics. *Deficit Therapy*.

[16] Feissel M., Michard F., Faller J. P., Teboul J. L. (2004). The respiratory variation in inferior vena cava diameter as a guide to fluid therapy. *Intensive Care Medicine*.

[17] Chen L., Hsiao A., Langhan M., Riera A., Santucci K. A. (2010). Use of bedside ultrasound to assess degree of dehydration in children with gastroenteritis. *Academic Emergency Medicine*.

[18] Schefold J. C., Storm C., Bercker S. (2010). Inferior vena cava diameter correlates with invasive hemodynamic measures in mechanically ventilated intensive care unit patients with sepsis. *Journal of Emergency Medicine*.

[19] Chen L., Kim Y., Santucci K. A. (2007). Use of ultrasound measurement of the inferior vena cava diameter as an objective tool in the assessment of children with clinical dehydration. *Academic Emergency Medicine*.

[20] Williams E. S., Shah S. J., Ali S., Na B. Y., Schiller N. B., Whooley M. A. (2008). C-reactive protein, diastolic dysfunction, and risk of heart failure in patients with coronary disease: heart and Soul Study. *European Journal of Heart Failure*.

[21] Kim J. H., Kim W. Y., Oh J., Kang H., Lim T. H., Ko B. S. (2020). Association of inferior vena cava diameter ratio measured on computed tomography scans with the outcome of patients with septic shock. *Medicine (Baltimore)*.

[22] Long E., Duke T., Oakley E., O’Brien A., Sheridan B., Babl F. E. (2018). Does respiratory variation of inferior vena cava diameter predict fluid responsiveness in spontaneously ventilating children with sepsis. *Emergency Medicine Australasia*.

[23] Mohammadpour M., Babaie S., Behzad A., Reisi M. (2018). A comparison between the bedside sonographic measurements of the inferior vena cava indices and the central venous pressure while assessing the decreased intravascular volume in children. *Advanced Biomedical Research*.

[24] Durajska K., Januszkiewicz E., Szmygel Ł, Kosiak W (2014). Współczynnik żyła główna dolna/aorta w ocenie nawodnienia – porównawcza ocena wyników pomiarów doświadczonych i niedoświadczonych badaczy w grupie młodych dorosłych. *J Ultrason*.

